# Activation of PTEN/P13K/AKT Signaling Pathway by miRNA-124-3p-Loaded Nanoparticles to Regulate Oxidative Stress Attenuates Cardiomyocyte Regulation and Myocardial Injury

This article has been retracted.

**DOI:** 10.1155/2022/8428596

**Published:** 2022-10-11

**Authors:** Yuan Cheng, Qing He, Na Li, Mengdi Luo

**Affiliations:** ^1^Key Laboratory of Advanced Technologies of Materials, Ministry of Education, School of Materials Science and Engineering, Southwest Jiaotong University, Chengdu 610031, China; ^2^Clinical College of Southwest Jiao Tong University, Chengdu, China

## Abstract

As a common cardiovascular disease, acute myocardial infarction seriously affects the health and life of patients. miRNAs play an important role in acute myocardial infarction. Based on miRNA obtained from the previous sequencing, this study investigated whether miRNA (miR)-124-3p-loaded nanoparticles (NPs) affect the phenotype of the acute myocardial infarction (AMI) rat. Nano-miR-124-3p decreased the myocardial infarction area, improved the myocardial tissue structure, and increased the degree of fibrosis. Nano-miR-124-3p decreased apoptosis and the expression of cleaved caspase 3, indicating its role in protecting and repairing the myocardium. To further verify the action mechanism of miRNA, a potential target gene of miR-124-3p, PTEN was identified by STARBASE and further confirmed using double luciferase assays. Following cotransfection of nano-miR-124-3p and PTEN, the areas of tissue structure damage, myocardial infarction, and fibrosis were substantially elevated. The expression of cleaved caspase 3 and the apoptosis rate in the nano-miR-124-3p and PTEN cotransfection group was also significantly increased. Bioinformatics analysis revealed that miRNA-124-3 may regulate oxidative stress injury by targeting PTEN. Taken together, miR-124-3p could protect and repair myocardial tissues through targeting PTEN.

## 1. Introduction

AMI is a common acute ischemic heart disease in clinics [1]. The morbidity and mortality rate of acute myocardial infarction due to chronic diseases is also gradually increasing [2]. Without timely diagnosis and treatment, it is very easy to miss the best treatment time, which seriously affects the patient's health and prognosis [3–5]. In recent years, miRNA has been widely proved to function as an important part in the occurrence and development of cardiovascular disease [6, 7]. miR-124-3p was identified as a potential regulatory candidate for AMI [8]. Inhibition of miR-124-3p expression reduced apoptosis by targeting the SIRT1-activated FGF21/CREB/PGC1*α* pathway and attenuating both inflammation response and oxidative stress in AMI rats [9]. In conclusion, miR-124-3p might be a target site for disease management to slow down the development of myocardial remodeling after AMI.

Biodegradable synthetic polymers are increasingly used in supportive therapy drug delivery devices [10]. As a synthetic polymer, poly (d,l-lactic-co-glycolic acid) (PLGA) could transport proteins [11], peptides [12], bacterial or viral DNA [13], and various anticancer drugs [14]. PLGA presents excellent biodegradability, biocompatibility, and sustained release [15]. PLGA particles overcome some of the limitations faced by current miRNA therapeutics. Although miR-124-3p has been identified functioning in AMI, there are currently no studies showing its effect in conjunction with PTEN. And nanoparticles have demonstrated in many studies that better therapeutic effects can be achieved through their delivery. Therefore, the aim of this study was to deliver miR-124-3p via PLGA nanoparticles to a rat model of myocardial infarction to explore how it regulates PTEN to act on myocardial tissue.

## 2. Materials and Methods

### 2.1. PLGA Nanoparticles Preparation

PLGA nanospheres were loaded with miR-124-3p and set a polymer solution at a concentration of 10%. Following the reaction between n-hydroxysuccinimide (NHS) and diethyl carbonate, methanol/Et2O (1 : 1) was added, centrifuged, and followed by abandoning the supernatant. PLGA-NHS ester was ultimately yielded after the pellet dried, which was then mixed with diisopropylethylamine and NH2-PEG-COOH (MW 3400) by dissolution. By the addition of MeOH/Et2O (1 : 1), the mixture was followed by two cycle washing, dried in vacuo, and gave PLGA-B-PEG-COOH. Cy5-conjugated miR-124-3p (Cy5/miR-124-3p) was supplied with DNase/RNase-free water and spermidine (15 : 1). The arginine-miR-124-3p complex was provided by dropwise to the obtained solution and sonicated at 40% amplitude with gentle stirring. The mixture was then treated using 5 ml of 1% PVA (w/v), gently stirred and followed by sonication under specified conditions to form a second emulsion. Finally, the enhanced nanoparticles were filtered, sterilized, and washed. miR-124-3p content was detected by a double-stranded DNA quantitative kit. Drug encapsulation efficiency (%) = measured amount of drug in nanoparticles/dosage (*μ*g/mg) × 100%. Drug loading (%) = nanoparticle drug content/total drug loading nanoparticles (*μ*g/mg) × 100% [16, 17].

### 2.2. Rat Model Construction for Myocardial Ischemia-Reperfusion

A total of 60 SD rats (male, six-eight weeks) were employed for constructing the model of rats. All were purchased from Chongqing Enswell Biotechnology Co., Ltd. The animals were anesthetized first to prepare for model construction. Here are the brief procedures during modeling: the rats were intubated after the removal of hair in the neck. The next step was to remove the hair in the chest, incise the skin on the left sternum edge, and open both third and fourth intercostal muscles to ensure a full exposure of the heart. Subsequently, a forceps was used to remove left atrial appendage (LAA) which was carefully lift up using a cotton swab. The vein between LAA and the lung cone was also visualized. The ligation marker could be positioned using the secondary vein. Suture 6-0 went through 1-2 mm from the left atrial root of the inferior coronary muscle to a depth of 2 mm. A double chain wire 2 was placed below the connecting wire. The surgical procedure was considered successful when the myocardium altered its color into dark red swiftly and turned white gradually. When ischemia occurred after ligation 30 min, reperfusion was formed by removing the suture to exhaust the air in the chest. Finally, the rats were administered with 80000 units of penicillin sodium.

### 2.3. Treatment of miR-124-3p

The rats were randomly administrated by injection with nano-NC agomir, nano-miR-124-3p agomir, nano-miR-124-3p agomir+NC-virus, and nano-miR-124-3p agomir+PTEN Lvx-virus in the tail vein 3 days after successful molding.

### 2.4. Triphenyl Tetrazolium Chloride (TTC) Staining

The animals were anesthetized with sodium pentobarbital and placed supine on a surgical bench. The heart was collected using a clean petri dish, and the heart was flushed with 0.9% saline into the aortic opening using a syringe to drain residual blood. The sections were placed in a 1% TTC solution, wrapped in tin foil to protect them from light and incubated at 37°C for 30 minutes. Following the removal of TTC staining solution, tissue samples were fixed and observed under a microscope, showing pale white in the infarcted area and purplish red in normal myocardial tissue. Infarct zone measurements: infarct zones (ISS) and ischemic zones (AARs) were calculated by IPP6.0 software.

### 2.5. HE Staining

Hematoxylin staining for 8-15minutes, rinse the excess dye with tap water. Differentiation with 1% hydrochloric acid and alcohol for the 30s and full washing with tap water for 10 minutes. Dye with 1% eosin solution for 10 min and rinse with tap water for 1 min. Then gradient alcohol dehydration, xylene transparent, and finally neutral gum seal, dry, and observe under the optical microscope.

### 2.6. Masson Staining

Tissue sections were subsequently prepared for masson staining. Firstly, the sections were stained with lapis lazuli blue staining, followed by Mayer hematoxylin staining and then differentiated using acidic ethanol differentiation solution. Following treated using aniline blue solution, the slices were dehydrated, hyalinized, and sealed with neutral resin.

### 2.7. TUNEL Assays

To determine apoptosis of sample cells, we subsequently perform TUNEL assays. The cells were fixed, washed, blocked, and incubated under appropriate conditions as per conventional operation procedures. Color development was performed for visualization.

### 2.8. mRNA Level Detection by qPCR

For qPCR detection, RNA was extracted first, then reverse transcription and quantitative detection were performed using Goldenstar™ RT6 cDNA Synthesis Kit Ver.2 and 2 × T5 Fast qPCR Mix (SYBR Green I), respectively. The primer sequences are as follows:

- miR-124-3p-FTGGCTGGACAGAGTTGTCAT
- miR-124-3p-RCTGTACAGGTGAGCGGATGTT
- PTEN-FACCAGGACCAGAGGAAACCT
- PTEN-RCCTTGTCATTATCCGCACGC
- GAPDH-F GCAAGTTCAACGGCACAG.
- GAPDH-R GCCAGTAGACTCCACGACATA.

### 2.9. Western Blot

Firstly, we performed total protein extraction to collect the supernatant. Total protein was mixed with SDS sample buffer, denatured by boiling, followed by SDS-PAGE seperation, PVDF membrane transferrence, and membrane blocking using 5% skim milk. Subsequently, incubation was performed at appropriate concentrations of primary antibodies cleaved caspase 3 (China, ABclonal, A19654), PTEN (China, ABclonal, A19104), P13K (China, abcam, ab182651), AKT (China, abcam, ab38449), and *β*-actin (China, ABclonal, AC026) at 4°C overnight. Secondary antibodies were also supplied. Finally, the enhanced chemiluminescence (ECL) detection reagent was used to mix and evenly cover the entire film, and after 1 minute of reaction, it was placed in an exposure meter for exposure detection.

### 2.10. Lentivirus Packaging and Infection of Animal Models

We performed miR-124-3p and PTEN lentiviruse packaging. The rat model was injected 10^8^ unit virus in caudal vein, and samples were taken subsequently.

### 2.11. Target Gene Detection by Dual-Luciferase Assays

Briefly, PGL4.11-BASIC, the reporter gene vector was used for preparing PETN-WT-LUC2-RLUC and PETN-MUT-LUC2-RLUC, respectively. Working solution luciferase assay reagent II (Progema) was applied. The expression of the reporter genes was monitored, recorded accordingly, and used as internal value.

### 2.12. PPI Network and GO Enrichment Analysis

Data related to prostate cancer and oxidative stress were obtained from the database https://www.ncbi.nlm.nih.gov/geo/query/acc.cgi?acc=GSE180765; the online database STRING (http://string-db.org) was utilized for the analysis of protein-protein interaction. The obtained DEGs were subjected to gene ontology (GO) analysis with the help of the R software packages cluster Profiler, enrichplot, and ggplot2. Only pathways with both P and Q values less than 0.05 were considered significantly enriched.

## 3. Results

### 3.1. Establishment of the Myocardial Infarction Rat Model

Infarct areas were visualized by TTC staining in the model group (Figure 1(a)). Meanwhile, myocardial tissue structure damage and fibrosis were also marked increased in the model by HE and Masson staining (Figures 1(b) and 1(c)). Furthermore, apoptosis of the model cells was substantially elevated after TUNEL method (Figure 1(d)), and so did the expression of cleaved caspase 3 in the model group as per the results of western blot (Figure 1(e)).

### 3.2. Characterization of miRNA 124-3p/NC miRNA-Encapsulated PLGA NPs

The average size and zeta potential of NC miR-encapsulated PLGA nanoparticles were 137.2 ± 5.636 nm and -14.1 ± 1.300, respectively, and those of nano-miR-124-3p were 137.9 ± 6.007 nm and –13.8 ± 0.748 mV. A certain amount of nanoparticles was added to DMSO to destroy the nanoparticle structure and release miR-124-3p, and the content of miR-124-3p was detected using a double-stranded DNA quantitative kit. The encapsulation efficiency and drug loading efficiency of miR-124-3p in PLGA-PEG nanoparticles were 78.4% ± 1.497% and 4.9% ± 0.3%, respectively (Table 1).

### 3.3. Nano-miR-124-3p Repairs Damaged Myocardial Tissue

Based on previous studies, we identified the miRNA with significant differential expression as miR-124-3p, whose expression was markedly decreased in model compared to Sham (Figure 2(a)). To clarify whether miR-124-3p-loaded nanoparticles exert a regulatory function in myocardial infarction rats, we transfected cultured rats with miR-124-3p and nano-miR-124-3p. TTC staining showed that the transfected latter nanoparticles significantly reduced infarct size of the animals (Figure 2(b)). Finding of HE staining revealed that myocardial cells in model presented an irregular arrangement, there were more collagen fibers, and the myocardial transverse striation was seriously damaged, accompanied by inflammatory cell infiltration, but nano-miR-124-3p improved the myocardial tissue structure (Figure 2(c)). Masson staining showed that a large number of blue collagen fibers were deposited in the myocardial tissue of model group, and degrees of fibrosis were serious. Nano-miR-124-3p reduced myocardial fibrosis and tissue damage (Figure 2(d)). The apoptosis results of TUNEL were similar to the above findings: the nano-miR-124-3p decreased apoptosis of the cells (Figure 2(e)). Overall, miR-124-3p has protective and repair functions in the myocardium.

### 3.4. PTEN Is a Target Gene of miR-124-3p

STARBASE prediction of possible miR-124-3p target genes indicated that PTEN might be one of its target genes (Figure 3(a)). The double luciferase assay further confirmed the previous test result that PTEN acted as a target gene of miR-124-3p (Figure 3(b)). Both western blot (Figure 3(c)) and qPCR (Figure 3(d)) findings revealed that PTEN expression increased in model compared to Sham. After miR-124-3p overexpression, PTEN expression decreased substantially in samples with miR-124-3p agomir and antagomir. Inhibition of miR-124-3p expression markedly elevated PTEN levels. Meanwhile, both P13K and AKT expression was increased significantly following overexpression of miR-124-3p but declined greatly following inhibiting miR-124-3p (Figure 3(e)).

### 3.5. MiR-124-3p Alleviates Myocardial Infarction through PTEN

Through the myocardial infarction rat model cotransfected with nano-miR-124-3p agomir and PTEN group, it is proved that nano-miR-124-3p can protect and recover myocardial infarction by targeting PTEN. Cotransfection of nano-miR-124-3p and PTEN overexpression markedly elevated myocardial infarct size, structure injury, as well as fibrosis (Figures 4(a) and 4(c)). In addition, the apoptosis rate and the expression of cleaved caspase 3 in the nano-miR-124-3p and PTEN overexpression cotransfection group were also significantly higher than those in the nano-miR-124-3p group alone (Figure 4(d)). Collectively, miR-124-3p protected and repaired myocardial tissues by targeted inhibition of PTEN, whereas after overexpression of PTEN, it was proven that nano-miR-124-3p could not exert its protective function which might be hampered.

### 3.6. miRNA-124-3p May Regulate Oxidative Stress Injury by Targeting PTEN

Myocardial cell injury occurs in myocardial tissue after ischemia-reperfusion injury, and oxidative stress also links to myocardial damage expansion during myocardial ischemia-reperfusion injury and has an association with acute myocardial infarction. To investigate whether miRNA-124-3p protects myocardial tissue by regulating oxidative stress injury, we screened 1223 differentially expressed genes for myocardial infarction and miR-124. GO enrichment analysis showed that these differentially expressed genes were involved in oxidative stress (Figure 5(a)). Strings screened 12 genes associated with PTEN (Figure 5(c)). Venn showed 3 genes at the intersection of the two mentioned above (Figure 5(b)). The chord diagram shows that TP53 genes in both intersecting sets link to the regulation of oxidative stress (Figure 5(d)).

## 4. Discussion

### 4.1. Successful Establishment of Myocardial Infarction Model of Rats

MI results from the blockage of the heart's own blood supply channels due to various factors [18]. With the change in people's lifestyles and the improvement of living standards, the incidence of acute myocardial infarction is increasing year by year. Acute myocardial infarction has a rapid onset and many complications, which seriously endanger human health [19]. Therefore, for acute myocardial infarction, early diagnosis and treatment are particularly important, which can improve the prognosis and improve the treatment effect. Postinfarction remodeling is largely dependent on infarct size [20, 21]. In this experiment, HE and Masson staining indicated an apparent damage in myocardial tissue structure of model rats and much worse myocardial fibrosis; the proportion of apoptotic cells and the expression of cleaved caspase 3 were also increased.

### 4.2. PLGA Nanoparticles Can Efficiently Deliver miR-124-3p

As a nonexpressed RNA, miRNAs are involved in the early development of the heart, and some miRNAs are only detectable in the heart, further confirming the value of miRNAs as cardiac markers [22, 23]. PLGA polymer nanoparticles can capture bioactive molecules and escape from cellular lysosomes into the cytoplasm, thereby inducing sustained release of intracellular transporters and prolonging the therapeutic effect. This study demonstrated that nano-miR-124-3p delivered via PLGA significantly reduced infarct size, improved myocardial tissue structure, and attenuated myocardial fibrosis. In addition, nano-miR-124-3p could significantly decrease apoptosis.

### 4.3. Nano-miR-124-3p Protects Myocardial Tissue by Targeting PTEN Inhibition

As a member of the miRNA family, miRNA-124-3p correlates with the proliferation and apoptosis of cells [24]. Multiple researches have indicated the great importance of miR-124-3p in cardiovascular diseases [25]. The PTEN gene is the first novel tumor suppressor gene with specific phosphatase activity that was cloned in 1997 and can effectively inhibit the growth of tumor cells [26]. The current research elucidated that the target gene of miR-124-3p PTEN mediated the progression of myocardial infarction. Cotransfection of nano-miR-124-3p and PTEN overexpression greatly enlarged the size of myocardial infarction, structure damage, and fibrosis. Apoptosis rate and the expression of cleaved caspase 3 were also much higher than those in the nano-miR-124-3p group, implying the protection function of nano-miR-124-3p in myocardial tissues via targeting the inhibition of PTEN, which did not work under the context of PTEN overexpression.

### 4.4. MiR-124-3 May Regulate Oxidative Stress Injury by Targeting PTEN

During myocardial ischemia, hypoxia occurs simultaneously and the body's ability to scavenge oxygen radicals is insufficient, while when reperfusion restores blood supply, a large amount of oxygen-rich blood flow rapidly enters the ischemic region in a short period of time, generating more cytotoxic substances such as oxidized radicals, causing cell damage, necrosis, or apoptosis [27, 28]. Reducing the formation of oxygen free radicals is beneficial to reducing apoptosis, mitigating myocardial injury, and improving myocardial function [29]. During AMI, reduced myocardial antioxidant capacity, increased oxidative stress, and increased cardiomyocyte apoptosis were observed [30]. Studies have shown that miR-340-5p protected cardiomyocyte apoptosis and oxidative stress induced by hypoxia and reoxygenation by regulating the Act1/NF-*κ*B signaling pathway [31]. miR-223-3p and miR-210 are also involved in oxidative stress injury and apoptosis in cardiomyocytes [32, 33]. In this study, bioinformatics analysis revealed that miRNA-124-3 may regulate oxidative stress injury by targeting PTEN.

## 5. Conclusion

This study demonstrates that PLGA nanoparticles can effectively deliver miR-124-3p to a rat model of myocardial infarction so that it can protect and repair myocardial tissue in myocardial infarction. Furthermore, it also reveals that nano-miR-124-3p protects myocardial tissue via regulating the PTEN/PI3K/AKT signaling pathway. This study confirms the role of miR-124-3p in myocardial injury, and it is expected to offer some directions for the management against this disease clinically.

## Figures and Tables

**Figure 1:** Histological examination of rats with myocardial infarction. (a) Myocardial infarct size was determined by TTC staining. (b) HE staining. (c) Masson stainings. (d) TUNEL staining. (e) Western blot of cleaved caspase 3 expression.

**Figure 2:** Protection and restoration of myocardial tissue by nano-miR-124-3p. (a) qPCR detection of miR-124-3p expression. (b) TTC staining. (c) HE staining. (d) Masson staining. (e) TUNEL staining.

**Figure 3:** Prediction and detection of PTEN being a target gene of miR-124-3p. (a) Prediction results of PTEN for miR-124-3p via STARBASE database. (b) The relative luciferase activity illustration using double luciferase assay. PTEN expression in both model and Sham groups were detected by western blot (c) and qPCR (d), respectively. (e) Detection of PTEN, P-P13K, and P-AKT expression by western blot after overexpression and inhibition of miR-124-3p.

**Figure 4:** Protection and restoration effects of nano-miR-124-3p on damaged myocardial tissue via targeting PTEN. (a) TTC staining. (b) HE staining. (c) Masson staining. (d) TUNEL staining. (e) Detection of cleaved caspase 3 expression by western blot after overexpression of nano-miR-124-3p and coexpression of nano-miR-124-3p and PTEN.

**Figure 5:** miRNA-124-3p may regulate oxidative stress injury by targeting PTEN. (a) GO enrichment. (b) Venn. (c) PPI. (d) Chord diagram.

**Table 1:** Characterization of miRNA 124-3p/NC miRNA-encapsulated PLGA NPs.

Group	Particle size (nm)	Zeta potential (mV)	Encapsulation rate (%)	Drug loading (%)
Nano-NC	137.2 ± 5.64	−14.1 ± 1.30	80.2 ± 2.04	4.9 ± 0.10
Nano-miR-124-3p	137.9 ± 6.01	−13.8 ± 0.75	78.4 ± 1.50	4.9 ± 0.30

## Data Availability

The data used to support the findings of this study are included within the article.
